The article "Risk Factors of Urinary Pathogenic Bacteria Infection after Benign Prostatic Hyperplasia Surgery and Curative Effect Analysis of Shuangdong Capsule Intervention" was retracted in 2024. Reasons: signs of a paper mill; suspected computer-generated content; unreliable results or conclusions; concerns about the data.

# Risk Factors of Urinary Pathogenic Bacteria Infection after Benign Prostatic Hyperplasia Surgery and Curative Effect Analysis of Shuangdong Capsule Intervention

**DOI:** 10.1155/2022/4069787

**Published:** 2022-09-08

**Authors:** Bing Xu, Ming Liu, Yonghui Liu, Jianhong Zuo

**Affiliations:** ^1^The Third Affiliated Hospital, Department of Urology Surgery, Hengyang Medical School, University of South China, Hengyang, Hunan 421900, China; ^2^The Third Affiliated Hospital, Department of Oncology, Hengyang Medical School, University of South China, Hengyang, Hunan 421900, China

## Abstract

Benign prostatic hyperplasia (BPH) is a common and frequently occurring disease in clinics, with the main manifestations including frequent micturition, urinary incontinence, dysuria, and endless urination. Transurethral resection of the prostate (TURP) is the main treatment for BPH, but some patients are prone to urinary tract infection after surgery, which affects the prognosis. Therefore, it is of great significance to study the pathogenic characteristics and risk factors of postoperative urinary-derived pathogenic bacteria infection in patients with BPH for the prevention and treatment of postoperative infection. In addition, the treatment of patients with this disease is also the focus of clinical attention. Long-term massive application of antibiotics can induce drug-resistant mutations of bacteria, so it is urgent to find an efficient and safe therapeutic scheme in clinics. However, traditional Chinese medicine (TCM) has a long history of treating urinary tract infections. Therefore, Shuangdong capsule, a traditional Chinese medicine preparation, was selected for the combined treatment in this study. The results showed that age, concomitant diabetes mellitus, and preoperative prophylactic application of antibiotics were the independent risk factors for postoperative urine-derived pathogenic infection in BPH patients. Clinical intervention for BPH patients with concomitant risk factors should be emphasized in clinical practice. The combined use of Shuangdong capsule and conventional western medicine can improve the clinical symptoms and inflammatory reactions of postoperative urine-derived pathogenic infection in BPH patients. Due to its exact curative effect and high safety, it is worthy of promotion. The clinical study registration number is M2022019.

## 1. Introduction

Benign prostatic hyperplasia (BPH) is a common male disease in the clinic and occurs more frequently in the middle-aged and elderly [1]. There are no typical symptoms of BPH in the early stage due to the compensatory effect of the body. However, with the progression of the disease, BPH can aggravate the degree of urinary obstruction, resulting in frequent micturition, urinary incontinence, dysuria, and endless urination [2]. Currently, patients with BPH are mainly treated with transurethral resection of the prostate (TURP). Although the clinical effect of TURP is very obvious, some patients are prone to urinary-derived infection after surgery under the influence of advanced age, concomitant underlying diseases, and other factors [3].

The article "Risk Factors of Urinary Pathogenic Bacteria Infection after Benign Prostatic Hyperplasia Surgery and Curative Effect Analysis of Shuangdong Capsule Intervention" was retracted in 2024. Reasons: signs of a paper mill; suspected computer-generated content; unreliable results or conclusions; concerns about the data.

Antibiotics are mainly used in the treatment of urinary tract infection after BPH operation in western medicine [4]. However, with the extensive use of antimicrobial agents in clinical practice in recent years, some pathogenic bacteria have developed strong resistance to conventional antimicrobial agents, which brings certain difficulties to the treatment of urinary tract infections [5]. In order to improve the clinical treatment effect and reduce the treatment efficacy of patients, the related research subsequently changed its research direction and further explored the field of traditional Chinese medicine [6]. TCM believes that urinary tract infection falls into the category of “stranguria,” mainly caused by damp-heat stagnation. Shuangdong capsule has the effects of clearing heat and stranguria, replenishing qi, and nourishing yin, which has the ideal clinical curative effect on alleviating or relieving the damp-heat in lower energizer and deficiency of both qi and yin [7]. Shuangdong capsule is mainly used to reduce or relieve the symptoms of frequent micturition, urgent urination, burning and stabbing pain in the urethra, and yellow urination caused by acute mild and moderate simple lower urinary tract infection [8]. However, few studies have reported the efficacy of this drug in the treatment of urinary tract infection after TURP. In this study, we analyzed the urinary pathogenic bacteria infection and risk factors in patients with BPH after surgery and further explored the efficacy of Shuangdong capsule intervention, in order to provide a basis for the prevention and treatment of postoperative urinary infection. The results are now reported as follows.

## 2. Materials and Methods

### 2.1. General Information

A total of 92 patients with BPH who received surgical treatment in our hospital from January 2022 to May 2022 were selected as the research subjects. Their ages were from 47 to 75 years, and the average age was (69.74 ± 10.33) years. The course of disease was from 2 to 15 years, with an average course of (9.35 ± 2.24) years. The volume of the prostate was 35 to 90 cm^3^, with an average of (58.64 ± 12.39) cm^3^. The preoperative International Prostate Symptom Score (IPSS) was 19 to 30 points, with an average score of (23.13 ± 3.15) score.

The article "Risk Factors of Urinary Pathogenic Bacteria Infection after Benign Prostatic Hyperplasia Surgery and Curative Effect Analysis of Shuangdong Capsule Intervention" was retracted in 2024. Reasons: signs of a paper mill; suspected computer-generated content; unreliable results or conclusions; concerns about the data.

### 2.2. Inclusion Criteria

Inclusion criteria were as follows: ① All of them had the main symptoms of frequent micturition, urgent urination, nocturia, and dysuria and were confirmed as BPH by color Doppler ultrasound and cystoscope tests. ② Patients with indications for transurethral resection of the prostate and undergoing surgical treatment, specifically including those with no improvement after regular drug treatment; patients with BPH with residual urine more than 50 ml measured by B-ultrasound; residual urine increased due to prostatic hyperplasia, repeated urinary tract infections, and bladder stones formed due to excessive residual urine; patients with urinary retention, etc. ③ There was no infection before operation. ④ There was no history of drug allergy. ⑤ This study was approved by the Medical Ethics Committee of the hospital. The patients and their families knew the situation and signed the informed consent form.

### 2.3. Exclusion Criteria

Exclusion criteria were as follows: ① patients with prostate cancer or reproductive tract cancer; ② those with diseases such as urinary system deformity, obstruction, and tumor discovered through B-scan ultrasonography or relevant examinations in the medical history; ③ those accompanied with bladder calculi; ④ patients with a history of urethral surgery before entering the group; ⑤ patients with incomplete clinical data and follow-up data.

### 2.4. Pathogen Culture and Identification

The infection status of urine-derived pathogenic bacteria after prostatectomy was counted. The urine samples collected from the patients in the middle stage of prostatectomy were sampled, separated, and cultured, and the strains were identified using ATB microbiological assay device manufactured by French BioMeria.

### 2.5. Collection of Baseline Information

Clinical data of all patients were collected through electronic medical records: ① general information: age, course of the disease, BMI, prostate volume, and IPSS score; ② combined basic conditions: diabetes mellitus, hypertension, and coronary heart disease; ③ surgical conditions: whether the urethral catheterization was conducted before the operation, the operation time, and the time of indwelling catheter after the operation; prophylactic application of antibiotics before surgery.

### 2.6. Treatment Methods

Patients after surgery were divided into control group and study group according to different treatment methods. Levofloxacin was used in the basic treatment in control group (Changchun Serene Pharmaceutical Co., Ltd., GuoYaoZhunZi H20203307, specification: 0.5 g). Oral administration: 200 mg/time, 3 times/d. On this basis, the research group orally took Shuangdong capsule (produced by Guizhou Remote Pharmaceutical Co., Ltd., GuoYaoZhunZi Z20120030, with the specification of 0.30 g/granule). Oral administration: 3 capsules/time, 3 times/day. Patients in both groups received medication continuously for 10 d.

The article "Risk Factors of Urinary Pathogenic Bacteria Infection after Benign Prostatic Hyperplasia Surgery and Curative Effect Analysis of Shuangdong Capsule Intervention" was retracted in 2024. Reasons: signs of a paper mill; suspected computer-generated content; unreliable results or conclusions; concerns about the data.

### 2.7. Observation Indicators

1. Clinical efficacy: the efficacy was evaluated according to the symptom score in traditional Chinese medicine (TCM). Symptoms included frequent urination, burning, and painful urination, dripping wet and unsmooth urination, abdominal distension, and pain due to limited appetite; Secondary symptoms included soreness of waist, low grade fever, distension of lower abdomen, bitter and dry mouth, emotional disturbance, constipation, red tongue, white or slightly greasy coating, and wiry and rapid pulse. The main symptoms were classified as asymptomatic (0 point), mild (2 points), moderate (4 points), and severe (6 points). For secondary symptoms, no symptoms indicated 0 points, mild 1 points, moderate 2 points, and severe 3 points. After treatment, the clinical symptoms and physical signs completely disappeared and the syndrome score decreased by more than 90% as compared with that before treatment meant recovery. After treatment, the symptoms and physical signs were significantly improved, and the decrease of syndrome score by 70%–89% as compared with that before treatment was considered as marked effect. Symptoms and physical signs were improved after treatment, and reduction of syndrome score by 30%–69% was considered effective. If there is no significant improvement in symptoms and physical signs after treatment and the syndrome score is less than 30% lower than that before treatment, it is considered ineffective [9]. Total effective rate = recovery rate + marked effective rate + effective rate.
2. Urine sediment leukocytes: mid-morning urine was taken in the morning, the urine samples were inoculated on blood agar plates with a quantitative inoculation ring, and the plates were placed in a 37°C greenhouse incubator for cultivation for 24 h; then, we take out the plate and count the number of colonies. Positive criteria: the number of bacteria in the clean midsection urine discharged from the urethra should not exceed 1 × 10^3^ CFU/mL [10].
3. Serum inflammatory factors: five milliliters of venous blood were collected from patients in the study group before and after treatment in a vacuum blood collection tube containing anticoagulant (K2-EDTA). After thorough mixing, the levels of serum-*α* (tumor necrosis factor (TNF, TNF-*α*), interleukin-6 (IL-6), and procalcitonin (PCT) were determined by enzyme-linked immunosorbent assay (ELISA). The detection steps included dilution, incubation after the addition of horseradish peroxidase, plate washing, addition of substrates *A* and *B*, incubation in the dark, addition of stop solution, and determination of OD value at a wavelength of 450 nm.
4. Adverse reactions: the drug-related adverse reactions observed in the patients during the treatment were recorded in details, including abdominal pain, diarrhea, and dry mouth.

The article "Risk Factors of Urinary Pathogenic Bacteria Infection after Benign Prostatic Hyperplasia Surgery and Curative Effect Analysis of Shuangdong Capsule Intervention" was retracted in 2024. Reasons: signs of a paper mill; suspected computer-generated content; unreliable results or conclusions; concerns about the data.

### 2.8. Statistical Methods

SPSS22.0 software was used for processing. The continuous variable data of experimental data were expressed as mean standard deviation ($\bar{x}$ ± *s*) and adopted *t*-test. The classified variable data and descriptive analysis were expressed as (%) and adopted *χ*^*2*^ test. A multivariate logistic regression model was used to analyze the significant factors in single factor analysis. The test level was *α* = 0.05, and *P* < 0.05 indicated that the difference was significant.

## 3. Results

### 3.1. Univariate Analysis of Postoperative Urinary Pathogenic Bacteria Infection in Patients with BPH

Forty of 92 BPH patients (43.48%) developed urinary pathogenic bacteria infection after the operation.

Univariate analysis showed that there was no significant difference in BMI, course of the disease, IPSS, concomitanthypertension, and intraoperative blood loss between the infected group and the noninfected group (*P* > 0.05). Age, prostate volume, concomitant diabetes mellitus, preoperative prophylactic application of antibiotics, preoperative catheterization, operation time, and postoperative indwelling catheter time were the single factors affecting postoperative urine-derived pathogenic bacteria infection in BPH patients (*P* < 0.05, Table 1).

### 3.2. Variable Assignment

The risk of infection was taken as a dependent variable, and the factors with significant differences in Table 1 were taken as independent variables to be included in the logistic regression model. The assignments of the dependent variable and independent variable are shown in Table 2.

### 3.3. Analysis of Multiple Factors Affecting Postoperative Urinary-Derived Pathogenic Bacteria Infection in Patients with BPH

Multivariate analysis showed that age, concomitant diabetes mellitus, and preoperative prophylactic application of antibiotics were the independent risk factors for postoperative urine-derived pathogenic infection in BPH patients (*P* < 0.05, Table 3).

### 3.4. Urine-Derived Pathogenic Bacteria Infection and Distribution in BPH Patients after Operation

A total of 76 pathogenic bacteria were isolated from 40 urine samples as shown in Table 4, including 43 Gram-negative bacteria (56.58%), 29 Gram-positive bacteria (38.16%), and 4 fungi (5.26%).

The article "Risk Factors of Urinary Pathogenic Bacteria Infection after Benign Prostatic Hyperplasia Surgery and Curative Effect Analysis of Shuangdong Capsule Intervention" was retracted in 2024. Reasons: signs of a paper mill; suspected computer-generated content; unreliable results or conclusions; concerns about the data.

### 3.5. Comparison of Clinical Effects of Patients with Different Treatment Methods

The total clinical effective rate of patients in the research group was significantly higher than that in the control group (*P* < 0.05, Table 5).

### 3.6. Comparison of Urinary Leukocytes and Serum Inflammatory Factors in Patients with Different Treatment Methods before and after Treatment

There was no significant difference in the levels of urinary leukocytes and serum inflammatory factors between the two groups before treatment (*P* > 0.05). After the treatment, the levels of urinary leukocyte, TNF-*α*, IL-6, and PCT in the research group of patients were lower than those before treatment and the levels of various indicators in the research group were lower than those in the control group (*P* < 0.05, Table 6).

### 3.7. Comparison of the Safety of Different Treatment Methods

No drug-related adverse reactions were observed in the two groups during the treatment.

## 4. Discussion

At present, the incidence of BPH increases year by year with the aging of the global population [11]. Surgical treatment is the main method for clinical treatment of BPH. However, patients are prone to postoperative infectious complications such as incision infection and urethral infection, which affects the recovery of patients [12]. Therefore, exploring the pathogen distribution and risk factors of postoperative urinary tract infection in patients with benign prostatic hyperplasia and formulating an effective prevention and treatment plan based on the pathogen distribution is conducive to taking targeted measures to prevent and treat urinary tract infection in the clinic.

The results of this study showed that the infection rate in 92 patients with BPH was 43.48% and the incidence of urinary tract infection was similar to the results of the previous study. It can be seen that patients with BPH have a higher probability of urinary tract infection after surgery. In this study, we found that age, concomitant diabetes mellitus, and preoperative preventive application of antibiotics were independent risk factors for postoperative urinary-derived pathogenic bacteria infection in BPH patients (*P* < 0.05). Based on previous studies, we analyzed the causes and further discussed the prevention strategies. ① For older patients, the immune system function is degraded, the tolerance to surgical trauma is reduced, and the possibility of bacterial invasion is increased [13]. At the same time, anesthesia will also break the normal environment in the body and reduce the body's immune function [14]. Therefore, elderly patients after surgery are often more prone to urinary tract infections. This suggests that clinical attention should be paid to elderly patients with BPH to prevent postoperative infection by strengthening nutrition before the operation, controlling basic diseases, and strengthening nursing after the operation. ② Patients with diabetes mellitus have their metabolic disorders, and the number of white blood cells with anti-infection function in the urine is significantly reduced. In addition, the high glucose environment provides a suitable environment and sufficient energy for the growth and reproduction of pathogenic bacteria, thus increasing the risk of postoperative urinary tract infection [15]. Therefore, clinical attention should be focused on patients with BPH with diabetes. The preoperative blood glucose was controlled by strengthening nursing intervention, strictly controlling diet, and combining with hypoglycemic drugs, to regulate the metabolic balance in the body. All of which increase the risk of postoperative urinary tract infection. ③ Prophylactic application of antibiotics before surgery can reduce postoperative urinary tract infection, which may be related to the effective control of asymptomatic bacteriuria with antibiotics before surgery [16]. Some studies have shown that asymptomatic bacteriuria can cause urinary tract infection, so it is extremely important to effectively control it before surgery [17]. In addition, previous studies have pointed out that preoperative urethral catheterization and postoperative indwelling urinary catheter for more than 7 d are also risk factors for postoperative urinary tract infection in BPH patients [18]. However, in this study, both of them were only a single factor affecting postoperative urinary tract infection in patients with BPH, and multivariate analysis showed that both *P* values were higher than 0.05. The reason may be related to the following aspects: On the one hand, before surgery, we paid attention to the evaluation of patient's clinical characteristics and strictly controlled the operation of preoperative catheterization and postoperative indwelling urinary catheter. On the other hand, our hospital strengthened the nursing intervention of various invasive operations and strictly controlled the aseptic operation, thus effectively preventing the occurrence of infection.

The article "Risk Factors of Urinary Pathogenic Bacteria Infection after Benign Prostatic Hyperplasia Surgery and Curative Effect Analysis of Shuangdong Capsule Intervention" was retracted in 2024. Reasons: signs of a paper mill; suspected computer-generated content; unreliable results or conclusions; concerns about the data.

In addition, the study believes that targeted treatment according to the results of its drug sensitivity test can improve clinical efficacy. In this study, a total of 76 pathogenic bacteria were isolated from the urine samples of infected patients, and only four fungi were found, with the rest being bacteria. This result confirmed that bacterial infection remained the main pathogenic species of postoperative urinary tract infection. Further analysis showed that *Escherichia coli* had the highest detection rate. As a type of opportunistic pathogens, it generally existed in the urinary tract and intestinal tract. However, patients with BPH had obstructed urethra, and urine retention could not be ruled out to increase the probability of infection. At the same time, the body was in a sterile environment under normal conditions. However, in elderly patients with decreased body function, urethral catheterization before surgery might destroy the inherent defense function of the urinary system, resulting in decreased resistance of urethral mucosa to pathogenic bacteria, leading to urinary tract infection [19]. Therefore, antibacterial drugs are mainly used for clinical treatment of postoperative urinary-derived infection. However, antibacterial drugs can effectively kill bacteria, but at the same time, they can cause damage to normal cells. In addition, with the increasing abuse of antibacterial drugs, the types of drug-resistant strains are increasing, and even there are many super-resistant bacteria and multiresistant bacteria. The effect of antibacterial drugs on urinary tract infection is also declining [20]. On account of this, commonly used clinical antibacterial drugs were used as the control drugs in this study to investigate the value of the combined treatment of traditional Chinese and Western medicine in the treatment of urinary tract infection.

Urinary tract infection falls into the category of “stranguria” in TCM. In TCM, stranguria is considered that starts from the invasion of the damp-heat pathogen into the lower energizer, with the dampness sticky and persistent. In addition, heat pathogen is likely to consume qi and hurt yin, as well as the deficiency of the spleen and kidney. Hence, stranguria is mostly a syndrome of deficiency-excess in complexity [21]. Therefore, in clinical treatment of stranguria, the deficiency-excess treatment should be combined, with the emphasis on exorcising pathogenic factors as well as strengthening vital qi [22]. Shuangdong capsule is prepared from Fructus Gardeniae, Radix Astragali seu Hedysari, Herba Hedyotis, Radix Ophiopogonis, Ramulus Et Folium Picrasmae, and Fructus Malvae. Gardenia and Hedyotis are bitter and cold, both of which are capable of clearing heat and removing dampness. In particular, Gardenia can clear the heat of the triple energizer in the human body and has the effect of diuresis. It can eliminate the dampness-heat pathogen from childhood and give the pathogen a way out [23]. The bitter and cold wood has the effect of clearing heat and drying dampness. Clinical pharmacology has also proved that the bitter wood has a strong inhibitory effect on *E. coli*. Modern pharmacology has proved that *Abelmoschus manihot* fruit has a significant role in promoting urination, which can make the damp-heat pathogen emerge from the feces and has a significant anti-inflammatory effect [24]. At the same time, Radix Astragali and Radix Ophiopogonis can help healthy qi and enhance the body's immunity to the etiology of both qi and yin deficiency. Radix Ophiopogonis is sweet and cold in nature, capable of nourishing yin and generating fluid, which is matched with Radix Astragali seu Hedysari to replenish qi and nourish yin. The results of this study showed that the total clinical effective rate in the research group was significantly higher than that in the control group. After the treatment, the levels of urinary leukocyte, TNF-*α*, IL-6, and PCT in patients of the study group were lower than those in the control group (*P* < 0.05), which confirmed that the combined use of Shuangdong capsule and conventional western medicine had exact therapeutic effect. It not only reduced the levels of urinary leukocyte and serum inflammatory factors, but also improved the clinical efficacy and symptoms of patients. In addition, there were no drug-related adverse reactions in the two groups during treatment, which also confirmed that taking Shuangdong capsule on the basis of levofloxacin was safe.

The article "Risk Factors of Urinary Pathogenic Bacteria Infection after Benign Prostatic Hyperplasia Surgery and Curative Effect Analysis of Shuangdong Capsule Intervention" was retracted in 2024. Reasons: signs of a paper mill; suspected computer-generated content; unreliable results or conclusions; concerns about the data.

In conclusion, the age, concomitant diabetes mellitus and preoperative prophylactic application of antibiotics were independent risk factors for postoperative urine-derived pathogenic infection in BPH patients. Clinical intervention for BPH patients with concomitant risk factors should be emphasized in clinical practice. The combined use of Shuangdong capsule and conventional western medicine can improve the clinical symptoms and inflammatory reactions of postoperative urine-derived pathogenic infection in BPH patients. Due to its exact curative effect and high safety, it is worthy of promotion. The deficiency of this study is that the sample sources are concentrated and the sample size is small, and the follow-up needs large-scale and multicenter research to further demonstrate the research results.

## Figures and Tables

**Table 1:** Univariate analysis of postoperative urinary pathogenic bacteria infection in patients with BPH.

Clinical features		Infected group (*n* = 40)	Noninfected group (*n* = 52)	*χ * ^*2*^/*t*	*P*
Age (years old)	<60	6 (15.00)	40 (76.92)	34.677	<0.001
	≥60	34 (85.00)	12 (23.08)		
BMI (Kg/m^2^)	<24	19 (47.50)	24 (46.15)	0.016	0.898
	≥24	21 (52.50)	28 (53.85)		
Course of disease (year)		9.42 ± 2.17	9.49 ± 2.19	0.154	0.879
IPSS (score)		24.18 ± 3.95	24.56 ± 3.71	0.475	0.636
Prostate volume (cm³)	<60	5 (12.50)	41 (78.85)	39.808	<0.001
	≥60	35 (87.50)	11 (21.15)		
Concomitant diabetes mellitus	No	7 (17.50)	42 (80.77)	36.356	<0.001
	Yes	33 (82.50)	10 (19.23)		
Concomitant hypertension	No	26 (65.00)	33 (63.46)	0.023	0.879
	Yes	14 (35.00)	19 (36.54)		
Concomitant coronary heart disease	No	25 (62.50)	30 (57.69)	0.217	0.641
	Yes	15 (37.50)	22 (42.31)		
Preoperative catheterization	No	9 (22.50)	20 (38.46)	5.655	0.017
	Yes	31 (77.50)	22 (42.31)		
Preoperative prophylactic application of antibiotics	No	32 (80.00)	16 (30.77)	21.960	<0.001
	Yes	8 (20.00)	36 (69.23)		
Operation time (min)	<60	11 (27.50)	44 (84.62)	30.676	<0.001
	≥60	29 (72.50)	8 (15.38)		
Intraoperative blood loss (ml)	<50	8 (20.00)	39 (75.00)	1.360	0.244
	≥50	32 (80.00)	13 (25.00)		
Postoperative indwelling catheter time (*d*)	<7	4 (10.00)	39 (75.00)	38.372	<0.001
	≥7	36 (90.00)	13 (25.00)		

The article "Risk Factors of Urinary Pathogenic Bacteria Infection after Benign Prostatic Hyperplasia Surgery and Curative Effect Analysis of Shuangdong Capsule Intervention" was retracted in 2024. Reasons: signs of a paper mill; suspected computer-generated content; unreliable results or conclusions; concerns about the data.

**Table 2:** Variable assignment of risk factors affecting postoperative urinary pathogenic bacteria infection in BPH patients.

Variable	Assignment
Dependent variable	
Infected	0 = no, 1 = yes
Independent variable	
Age	0 = <60 years old, 1 = ≥60 years old
Prostate volume	0 = <60 cm³, 1 = ≥60 cm³
Concomitant diabetes mellitus	0 = No, 1 = Yes
Preoperative catheterization	0 = No, 1 = Yes
Preoperative prophylactic application of antibiotics	0 = No, 1 = Yes
Operation time	0 = <60 min, 1 = ≥60 min
Postoperative indwelling catheter time	0 = <7 d, 1 = ≥7 d

**Table 3:** Analysis of multiple factors affecting postoperative urinary-derived pathogenic bacteria infection in patients with BPH.

Variable	*β*	SE	Wald *χ*^*2*^	*P*	OR	OR of 95% CI	
						Upper limit	Lower limit
Age	−3.728	1.866	3.990	0.046	0.024	0.001	0.932
Prostate volume	−4.179	2.035	4.215	0.040	0.015	0.000	0.828
Concomitant diabetes mellitus	−3.188	1.580	4.073	0.044	0.041	0.002	0.912
Preoperative catheterization	−2.172	1.596	1.853	0.173	0.114	0.005	2.599
Preoperative prophylactic application of antibiotics	−4.468	1.646	7.371	0.007	0.011	0.000	0.289
Operation time	−2.733	1.586	2.971	0.085	0.065	0.003	1.454
Postoperative indwelling catheter time	−1.758	1.744	1.017	0.313	0.172	0.006	5.257
Constant	12.996	4.401	8.722	0.003	814.701	—	—

**Table 4:** Urine-derived pathogenic bacteria infection and distribution in BPH patients after operation.

Pathogenic bacteria species		Plant number	Constituent ratio (%)
Gram-negative bacteria	*Escherichia coli*	28	36.84
	*Klebsiella pneumoniae*	15	19.74
	*Pseudomonas aeruginosa*	12	15.79
	Other	3	3.95
Gram-positive bacteria	*Enterococcus faecium*	13	17.11
	*Enterococcus faecalis*	10	13.16
	*Staphylococcus epidermidis*	5	6.58
	Other	1	1.32
Fungi	*Candida albicans*	3	3.95
	Other	1	1.32

The article "Risk Factors of Urinary Pathogenic Bacteria Infection after Benign Prostatic Hyperplasia Surgery and Curative Effect Analysis of Shuangdong Capsule Intervention" was retracted in 2024. Reasons: signs of a paper mill; suspected computer-generated content; unreliable results or conclusions; concerns about the data.

**Table 5:** Comparison of clinical effects of patients with different treatment methods.

Group	Recovery	Marked effective	Effective	Ineffective	Total effective rate (%)
Research group (*n* = 20)	16	5	1	1	95.00
Control group (*n* = 20)	8	4	2	6	70.00
*χ * ^*2*^			4.329		
*P*			0.037		

**Table 6:** Comparison of urinary leukocytes and serum inflammatory factors in patients with different treatment methods before and after treatment ($\bar{x}$ ± S).

Group	Urinary leukocyte		TNF-*α* (ng/L)		IL-6 (ng/L)		PCT (pg/L)	
	Before treatment	After treatment	Before treatment	After treatment	Before treatment	After treatment	Before treatment	After treatment
Research group (*n* = 20)	90.94 ± 25.83	32.15 ± 7.94^a^	25.33 ± 4.25	16.89 ± 2.91^a^	60.24 ± 12.36	38.91 ± 6.12^a^	159.24 ± 26.12	124.24 ± 20.61^a^
Control group (*n* = 20)	91.06 ± 25.57	20.38 ± 7.04^a^	25.06 ± 4.14	12.04 ± 2.01^a^	60.22 ± 12.71	29.24 ± 5.12^a^	159.32 ± 26.33	108.22 ± 21.45^a^
*t*	0.015	4.960	0.204	6.134	0.005	5.420	0.010	2.408
*P*	0.988	<0.001	0.840	<0.001	0.996	<0.001	0.992	0.021

*Note.* ^a^ *P* < 0.05, compared with that in the same group before treatment.

## Data Availability

The data used and/or analyzed during the current study are available from the corresponding author.
